# False Vision Graphics in Logo Design Based on Artificial Intelligence in the Visual Paradox Environment

**DOI:** 10.1155/2022/1832083

**Published:** 2022-09-13

**Authors:** Hexin Zheng

**Affiliations:** Zhongge School of Arts, Guangdong Ocean University, Zhanjiang 524088, China

## Abstract

There are numerous fresh ways of thinking and creativity as a result of the ongoing development of art design. How do you create a fantastic logo that has extraordinary artistic effects? The incorrect interpretation of artistic graphics can cause a special visual phenomenon known as the contradiction between visual images and objective reality, which causes people's visual systems to produce points of interest. Wrong vision graphics, or visual paradox, can give people a wonderful experience that transcends time and space and reveals the enigmatic beauty that is concealed in the natural order, which is in line with the design goals of sign art. The integration of design and artificial intelligence has drawn a lot of attention as science and technology have advanced. Designing an intelligent and comfortable user experience is more important than ever, especially given the world's growing digital demand. The technical limitations of algorithm black boxes exacerbate the power disparity between humans and algorithms, which is inherent in artificial algorithms. According to its research, artificial intelligence's algorithm is responsible for roughly 60% of its calculations. Random forest technology's current benefits and drawbacks are contrasted with those of popular algorithms, and a clear vision of its potential applications in the future is presented. The artificial algorithm's recommended operation mechanism chooses the algorithm's nontechnical neutrality and value orientation.

## 1. Introduction

Whether it is engineering design to find solutions to complex problems or artistic design of paintings and products, artificial intelligence and design exhibit good synergy under the general environment of AI. Artificial intelligence provides design with possibility and uncertainty, while design is given a fresh approach to problem-solving by artificial intelligence. With the continuous development of art design, there are many new ways of thinking and creativity. How to design an excellent logo and how to make the logo have extraordinary artistic effect has become a problem to be studied by graphic design professionals. Nowadays, it is an era of “visualization” and “picture reading.” People's eyes are full of diversified symbols and all-round graphics. Graphics have formed a way of expression that transcends language, and people can quickly read the meaning directly from the surface without language barriers. When the observer's subjective grasp is not completely consistent with the existence of the object, it leads to false vision. It will make the observer have hallucination thinking, thus strengthening the intensity of visual perception of things, resulting in visual errors between the part and the whole, showing a strong idea of changing things, and finally achieving the goal of experiencing beauty with self-desire. The structure of random forest decision tree is a kind of modeling with algorithm, and the voting before branches and leaves is used for decision analysis. Artificial algorithm, that is, the computer simulates people's thinking and intelligence, runs according to a set program under a certain input premise, and the computer completes the output of a specific function, the accurate description of the method to solve a specific problem or clear limited instructions. With the development of society, artificial intelligence is gradually known to people. Especially since the economic crisis in 2008, the United States, Japan, and Europe have placed their hopes on the reindustrialization of artificial intelligence such as robots. At this opportunity, artificial intelligence technology has continuously made breakthroughs in various fields, bringing convenience to people's daily life and production but also causing many ethical problems such as human rights. Artificial intelligence technology is being used more and more frequently in social production and life due to the rapid development of AI, which not only alters the industrial model but also improves the quality of human life [1]. Although the frontier and centre of science and technology in the twenty-first century is artificial intelligence, it will inevitably lead to a number of new issues, including ethical ones. The scope and depth of applications of artificial intelligence in social life are expanding with the advent of the third revolution in artificial intelligence, which is characterised by deep learning. Artificial intelligence now permeates nearly every aspect of modern society, including administration of justice, healthcare, education, security, and communication, and it is starting to replace humans in some routine and decision-making tasks [2].

As artificial intelligence research [3] and development enters a new phase, the public is increasingly focused on the functionality of these products and the state of scientific and technological advancement, while the ethical and social issues brought on by their use are given only secondary consideration. Cloud computing has been set up as the primary framework for artificial intelligence applications, and many businesses also store their own data there. People's privacy rights have been violated to varying degrees, and artificial intelligence will unavoidably “read out” many unspeakable secrets of human beings while deeply analyzing massive data through cloud computing. However, when people enjoy the convenience brought by artificial intelligence technology, they gradually start to worry. Whether artificial intelligence will develop beyond the control of human beings will pose a threat to the survival and development of human beings. One of the typical hypotheses is that super robots are out of the control of human beings and completely dominate the world, and human beings are controlled by them. The controller of artificial intelligence algorithm, relying on the data technology barrier of “algorithm black box,” uses the algorithm to influence the social preference and political preference of the audience and influences and manipulates the audience's behavior pattern imperceptibly.

This paper uses a variety of research methods to analyze and explain it. In the research of artificial intelligence, the corresponding calculation formula and model diagram are used and established to explain and analyze it. In the sign design of right and wrong images, the method of establishing data map is used to analyze and understand them.

The main contributions of this paper are as follows:

1. The multievidence method is employed in this paper to describe and evaluate its research
2. In this paper, the model diagram and data diagram are established to explain and analyze the results and arguments of the research
3. The purpose of this study is to examine the use of artificial intelligence in the logo design of false vision graphics in order to demonstrate that the decision based on artificial intelligence is currently the most promising one

The rest of this paper is arranged: the second part introduces and analyzes the related work. In the third part, the corresponding research and analysis are made on the logo design of false vision graphics. The fourth part makes corresponding research and analysis on artificial intelligence. The fifth part summarizes the full text.

## 2. Related Work

Strong artificial intelligence and super artificial intelligence, in particular, have altered not only the course of economic and social development but also the relationships between individuals, among themselves, and with nature. With the development of technology, so too has the ethical risk of its application and promotion. Research and development of humanoid robots with emotional capabilities are becoming increasingly sophisticated as artificial intelligence advances. As nannies, pets, lovers, and parents, they “participate” in human life. Over time, they will also develop a variety of emotional and interest entanglements. These events' occurrence will have various effects on interpersonal relationships, family relationships, and workplace relationships. The importance and value of engineering technology research and development in artificial intelligence are both socially significant. The first level is based on the core value of human social development, and the second level is based on the tool technology of social development. Both levels are indispensable, and only the research of engineering technology is bound to have social ethical risks. Artificial intelligence is the development trend of information technology, and intelligence is also an important feature of today's society. Like any technological change, the development and change of artificial intelligence technology also brings some risks, but its development is a double-edged sword, which has both negative and positive significance for human society. Artificial intelligence must be developed within the bounds of appropriate ethics in order to flourish. Science has no boundaries, but the ethics of science and technology have limits. While artificial intelligence has had positive effects on real-world situations recently, its negative effects have also garnered attention. Studying the ethical issues brought on by artificial intelligence technology can not only deepen our understanding of that technology but also aid in understanding artificial intelligence and its ethical issues, enrich our ethical thinking, even lead to the formation of new ethical principles, and provide fresh concepts and a theoretical framework for addressing the ethical issues brought on by that technology.

In the research, Mellir and Kalogirou think that the impact of technology on the ecological environment involves deep-seated issues such as ethics, morality, and value [4]. Kohavi believes that unless human intelligence can reach the limit, artificial intelligence can never really surpass human intelligence, so it is meaningless and unnecessary to discuss the replacement of human intelligence [5]. O'Leary believes that moral subject should be a subject with moral consciousness and engaging in moral activities [6]. Dewey et al. think that artificial intelligence is just a robot, and the application of artificial intelligence is limited to industry. Until the 21st century, people began to study the corresponding ethical issues related to artificial intelligence and human society and the various influences of artificial intelligence on human subject, security, interests, and environment [7]. Colin proposed that both humans and robots can abide by the same psychological laws. We should regard the robot as an artificial life or a machine. The decisive factor is not the scientific discovery, but the decision made by people. When the development of robot technology is perfect and mature, robots will take the initiative to ask for rights [8]. Putzolu et al. put forward an attempt to systematically and deeply expand the ethical issues of weak artificial intelligence, strong artificial intelligence, and super artificial intelligence and demonstrate the differences and historical and social nature of ethical issues in different stages of artificial intelligence development [9]. From the perspective of science and technology ethics and ecological ethics, this paper expounds the mechanism and ecological, compound, and diversified characteristics of ethical problems in the development of artificial intelligence and points out the uncertain ethical risks in the development of artificial intelligence. Zucker puts forward that morality is mainly formed by emotion, not created by reason, thus forming the viewpoint of emotionalism ethics. Even Kant, a pure rationalist, cannot deny the existence of emotion in morality and morality [10]. Ou puts forward that the application of artificial intelligence technology needs to achieve the principles of fairness, transparency, reliability, tolerance, responsibility, privacy, and so on [11]. Sun puts forward the obligation of data protection impact assessment, which requires the data controller to undertake the analysis, assessment, and control of data processing risks. The regulatory authorities only review the assessment report without participating in the specific assessment process [12].

## 3. Research on Logo Design of 3 Wrong Vision Graphics

### 3.1. The Application of False Vision Graphics in Logo Design

Optical illusion graphics are not only widely used in the field of graphic design but also gradually become an important way to enrich the means of product design. There are many kinds of illusion phenomena, such as assimilation, brightness change, shape distortion, map-ground inversion, dimension transformation, and angle designation. False vision design is not a new design technique; it is only a small part of three major components (plane component, color component, and three-dimensional component). In product design, no matter how to deal with plane or three-dimensional, we often encounter the phenomenon of optical illusion. There are many examples of applying optical illusion design, and proper application will produce good modeling effect. When people appreciate artwork with a strong visual impact, their attention frequently shifts from purely aesthetic attraction to a proactive investigation of the viewer's heart. Despite the flatness of the product drawing, the actual product has three dimensions. Between plane and stereo, there is a noticeable difference in how things feel, and there will be different perspective distortions as you lean, level, and look up. A unique law of vision governs perspective, just like illusion. People's eyes have an extremely similar structure to cameras. The human eye's function goes beyond just that, as the camera only responds physically to things directly, and the influence it takes in is also communicated to the brain as information in some other way. The pinnacle of people's spiritual endeavours has always been the creation of art. Art's importance lies in its ability to bridge disparate human emotions. Most artistic works convey to viewers a sense of beauty that is both understandable and indescribable. Algorithms and models in artificial intelligence are examples of this kind of creativity and innovation [13, 14]. Symbiosis refers to the fact that several objects form an inseparable whole with a unique close relationship by sharing parts or contours, borrowing from each other, and setting off each other. There are many techniques of modern logo design, including a large number of optical illusion techniques. The points of interest caused by these optical illusions attract designers and the public together. The public, while pursuing to solve the optical illusion, also increases their awareness and memory of the logo, which makes the logo play a better role in identifying and conveying information. Establish its model diagram for analysis in its design, as shown in Figures 1 and 2.

The desire for data analysis is where the concept of quantification originated. Design, as an inventive and scientific cross-discipline, is obviously unable to deal with the data because of the enormous volume and variety of data, despite the fact that there is still debate about how to quantify artistic and cultural resources. The traditional design process also involves a lot of repetitive work. The original bulky, dull, and stiff shape is transformed into a light, fine, and novel shape by using the law of optical illusion to enhance the modeling effect. Correcting the wrong vision entails using the wrong vision law as the foundation, fully estimating the wrong vision, and appropriately changing some quantities and some relationships in the actual design, so that the vision affected by the wrong vision can be “compensated” or “restored” into a normal effect. The inherent laws of human vision, which are revealed by false vision graphics, exist in physiology and psychology and are constant because of the differences of times and regions. Especially in the field of logo design, the logo graphics created by wrong vision have the aesthetic feeling beyond the cultural background and geographical limitations [15]. False vision sign is to make use of people's visual false vision principle to connect the impossible morphological structures in the display space into a whole, inadvertently changing the logical relationship of the natural space and the habitual perspective law of the morphological structures and creating an illusion effect that seems reasonable but is full of contradictions in essence. The formation of dimension transformation usually uses the transformation and alternation of viewpoints, which breaks people's habit of dealing with the required objects selectively and produces a dreamlike visual experience. In all kinds of visual fields [16], the dimension transformation method is the most widely and frequently used illusion technique. In the research, a data map is established to analyze and explain it, as shown in Figure 3.

An optical illusion created by mixing and misplacing the shapes of various dimensional spaces is known as the “mixed-dimensional optical illusion.” Mixed-dimensional optical illusions can be created in a variety of ways, including switching between a two-dimensional plane and a three-dimensional space and shifting the isomorphism of different spatial levels. The process of meeting user needs is also a part of design, which on the one hand shapes the image of the product. The society of today is wealthy in material resources, and technology is continually developing. Users' demands and expectations for design products have significantly changed from the conventional form of emphasis to the content and experience. As a result, usability and practicality are now more important from a design standpoint than the more traditional emphasis on an object's surface. A growing number of people are thinking about incorporating traditional cultural elements into fashion designs in order to better promote cultural heritage, thanks to the ongoing development of humanities and the arts. Fashion is no longer just some exaggerated and unique designs.

### 3.2. Research on the Influence of False Vision Graphics on Logo Design

Although illusion is interesting, it has not been widely used in contemporary design. Because we do not know the modeling techniques of right and wrong art, or we do not know other things deeply enough, it is inevitable that right and wrong art often turns a blind eye, let alone pay enough attention to its special functionality. Generally speaking, a picture with a contrast between reality and falsehood will make people feel that there is a relationship between distance and distance, the scenery is deep and shallow, and the sense of three-dimensional space is strong. In the graphics and image software, we can focus selectively at will, even if it is the same focal plane, and we can also make different virtual-real relationships and produce wrong visual space feelings through the light-shadow relationship that deviates from reality. Reasonable expression of optical illusion can make the sign form very decorative and interesting. With the mystery and particularity of optical illusion graphics, designers and audiences can have ideological resonance. The ingenious application of false vision graphics in logo design lies in the dislocation and splicing of visual contour lines, which mysteriously changes the usual link rules when expressing spatial forms. This paradox structure, which cannot be produced in reality, often has a confusing and absurd visual effect, which is a subversion of habitual visual experience. In the influence of its research, the data tables are established for further analysis and explanation, such as Tables 1 and 2.

Optical illusion is a special graphic language, and we should make proper use of it to create the visual sense of space in the form of signs. In the process of using optical illusion, we should pay attention to the grasp of “degree.” The application of right and wrong vision should consider not only the visual modeling elements but also the background elements. Only when the two elements reach a balance can the wrong vision become a phenomenon of “changing movement” by guiding the alternate movement of the line of sight, so as to strengthen the content. With the increase of information, simple graphics can no longer attract people's attention, and it is undoubtedly a good way to enhance the visual communication of graphics by effectively using false vision and increasing the interest of graphics.

## 4. Artificial Intelligence Research

### 4.1. Introduction and Algorithm of Artificial Intelligence

With the advent of computers in the 1950s, artificial intelligence technology entered history's stage for the first time, and people started studying it seriously at that time. Artificial intelligence research aims to make machines that can handle tasks that require intelligent processing take the place of humans and free them from complex work that has varying justifications over time. The development and use of artificial intelligence [17] products is currently on the rise, largely due to the large market potential and the ongoing progress of human science and technology. The continual popularisation and application of artificial intelligence technology will fundamentally alter human society's present and future way of life, greatly enrich its social options, and vastly increase its ability to produce and live in new areas [18, 19]. This is a choice that has been made necessary by the advancement of science and technology in recent years. Generally speaking, artificial intelligence is an artificial product, so its mechanical characteristics should be open and transparent. At present, we do not know to a great extent how the artificial intelligence system draws a certain conclusion through deep learning and other means. The decision-making process of artificial intelligence is an invisible “black box” to a considerable extent. Since the beginning of the third scientific and technological revolution, people's production and lifestyle have gradually changed, and human beings have entered the information age and intelligence age. High-tech industries have gradually become the driving force to promote social development, among which artificial intelligence is the most prominent. Facing the enterprises with data advantages and the capital forces behind artificial intelligence algorithms, to build the supervision and regulation system of artificial intelligence algorithms, we should first make use of the massive data held by administrative organs to build a big data artificial intelligence algorithm system led by administrative forces and strengthen the ability of providing public services. Its application principle is based on the algorithm of decision tree, and then through the fitting algorithm, the scattered decision trees are integrated. Each tree is built on an independent sample. The distribution of tree categories in random forest has commonality, and the classification of categories comes from the classification ability of monomer number and the correlation with it. The algorithm used for distinguishing features is based on random free combination of nodes [20]. According to its research method, the corresponding algorithm formulas are established for analysis.

(1) $$\begin{array}{c} k_{x}={\left|\bar{u^{1}},-t_{-u}^{\prime \prime }\right|}_{2}^{1}\nu , \end{array}$$

(2) $$\begin{array}{c} \left\{-1\left\|x-12∋\overset{-1}{\underset{x\cdot }{\sum }}i=0\right\|x=\gamma l\pi \right., \end{array}$$

(3) $$\begin{array}{c} \mathrm{grad}\frac{x}{-l_{z}^{\prime \prime }},{tr}^{\prime }F, \end{array}$$

(4) $$\begin{array}{c} -\left|\overset{⟶}{x}+\lambda \right|,{\left.\frac{-11}{2t}\right|}_{-2}^{1}L^{\prime \prime }, \end{array}$$

(5) $$\begin{array}{c} x+tR{\bar{\lambda }}_{C}^{\prime }=\partial v_{x}^{\prime }C_{1}. \end{array}$$

The random machine model of forest uses the random combination of decision trees to achieve the algorithm purpose. Decision tree is a hierarchical type structure. The features described by each point and surface node are different from those described by point and edge. In the era of artificial intelligence algorithms, the open source data characteristics of artificial intelligence algorithms make effective supervision difficult. Therefore, the government should rely on the construction of its own big data platform to get rid of the problems of data siltation caused by bureaucracy within the government, lack of effective data sharing among departments, and poor data interconnection among regions, so as to realize data interconnection and become a dominant position in the field of big data, and rely on this to ensure that the supervision of artificial intelligence algorithms developed by Internet giants is implemented. As far as the actual application effect of artificial intelligence technology is concerned, the application of this technology conforms to the development trend of human society and the historical trend of scientific and technological revolution. Artificial intelligence consists of two key words, namely, “artificial” and “intelligent.” Actually, labor is not difficult to understand. In the scientific community, although there are different ways of expression, the definition of labor can basically be unified, that is, individuals within the organizational framework work and run according to the prescribed procedures in advance, so as to give full play to the collective strength and achieve the expected results or functions. Simply put, everything is arranged manually. According to its research, the corresponding data analysis chart is established to analyze and explain it, as shown in Figures 4 and 5.

In the 1950s, a conference of academics at Dartmouth gave birth to the idea of artificial intelligence. Numerous academics have shared their own opinions and research on “artificial intelligence” since it was first proposed. The end results of human brainpower are all feedback products. The body produces actions and develops intelligence when the products are fed back to it continuously. The early studies of artificial intelligence were greatly influenced by this concept. The precise goals change frequently as artificial intelligence technology advances. The ultimate goal of artificial intelligence technology development, for instance, is for computers to learn by solving problems and gaining new experiences like people do and even to master the “jumping learning” of creation. Therefore, artificial intelligence technology will undoubtedly give human society a vigorous boost as it develops, and as a result, it will attract more public attention. Because of the technical challenges posed by the algorithm's “black box,” it is challenging to hold the algorithm accountable. In the future rule of law framework of artificial intelligence algorithm, the specific obligations of algorithm developers will be added, and the transparency requirement will be embedded in the algorithm design. At the same time, the concept of zero-knowledge proof will be introduced; that is, in some important decisions, decision-makers will be allowed to provide proof for the decision-making without disclosing the contents and policies of important factors. The random forest model has been proved to produce overfitting behavior in some categories or problems with large errors and indistinct identification. In the research, the corresponding algorithm formulas are established.

(6) $$\begin{array}{c} y+H^{-}⊢H_{-}^{x}-11F=\lambda +x, \end{array}$$

(7) $$\begin{array}{c} 1=x⟶\left(1,-1^{\lambda }x+1^{r}\right), \end{array}$$

(8) $$\begin{array}{c} \frac{x_{-.1}}{1-x-1}\overset{x-1}{\underset{x-1}{\sum }}i,\underset{-T^{x}}{\sup}1=\frac{1}{J}, \end{array}$$

(9) $$\begin{array}{c} t\times \left(v+1\right)+u+k\left(T+\tau^{\prime }\times 1^{\prime }\right), \end{array}$$

(10) $$\begin{array}{c} F_{x}+\underset{x^{\prime }}{res}+\frac{1}{x}h^{-}=\frac{p^{\prime }}{,1}. \end{array}$$

Based on the expected use, key types, and acceptable error types of the algorithm, it is proposed that the design, testing, and guiding algorithm development should meet the performance standard of safety margin. In addition, the artificial intelligence algorithm itself is in the process of continuous self-learning and upgrading, and its automatic decision-making steps are often updated after the algorithm machine learning or human manipulation, combined with new data. In this regard, even if the source code and data are mastered, it is difficult to restore the decision-making process of artificial intelligence algorithm. The advancement of artificial technology aims to create artificial systems with a certain level of intelligence, attempting to use computers to perform tasks that previously required human intelligence, i.e., to research how to use computer hardware and software to simulate some intelligent human behaviours. In order to make artificial intelligence even more useful, people study the solutions to multiobjective problems that involve multiple intelligent agents on the basis of studying distributed problems with the same goal and acknowledge that artificial intelligence algorithms are used in governance. In order to master data power and face the challenge posed by the strength of artificial intelligence algorithms under capital control, sort out the sedimentary data, summarise, sort, and analyze them, determine the data value contained in them, and build a big data platform for the construction of service-oriented government on this foundation.

### 4.2. Artificial Intelligence Application and Problem Research

The development of artificial intelligence technology is a cutting-edge field that relies on the establishment of collaborative relationships among numerous fields, including linguistics, psychology, information theory, cybernetics, computer science, and even philosophy. Its primary research objective is to develop and implement intelligent human behaviours using machines, primarily computers. It has seen success across many fields after decades of development and optimization. Diverse forms of artificial intelligence, such as small sweeping robots, powerful underwater extreme operation robots, and large cargo robots, have gradually developed to help people complete their tasks more quickly and effectively. This is due to the ongoing innovation in artificial intelligence technology. Using the decision tree function of random forest model, combined with knowledge map, a new intelligent audit mode is generated, which is deeply applied on the basis of the exploration of existing audit innovation. The audit clues are used to construct the audit knowledge map database by knowledge map technology. Through the map method, the frequent problems of audit samples are holographically displayed, and the root causes of the frequent problems are deeply expanded and grouped, so as to establish the first professional knowledge map of audit specialty and realize intelligent and accurate audit. The continuous innovation of science and technology has led to the fact that human beings are no longer subject to the natural environment and pay no attention to balanced development, which indirectly leads to the unlimited development of resources, while the utilization rate of resources fails to reach the expected goal, which directly leads to the waste of resources. In the process of resource exploitation, a lot of artificial intelligence beyond the reach of human can help people realize it. The rapid development of artificial technology, especially freight robots and palletizing robots, enables entrepreneurs to obtain greater profits with higher efficiency and lower cost in a short period of time, which greatly reduces the employment space of manual workers. The manual labor industry is also gradually transforming towards mechanization, intelligence, and high efficiency, accompanied by a substantial increase in the number of people engaged in mental work. According to its research, the corresponding data graphs are established to analyze and explain it, as shown in Figures 6 and 7.

The widespread use of artificial intelligence technology has established itself as an unstoppable trend, and the numerous ethical issues brought on by the application of this technology's ambiguous moral status have emerged as a significant barrier to the advancement of human society as a whole. Establishing artificial intelligence's moral subject status will help to ensure that when it injures the rights and interests of others or society through its use in technology, the accountable subject will be identified in due time, and the artificial intelligence will be urged to take on its proper responsibilities. The widespread use of artificial intelligence in many facets of society has become the norm as a result of society's quick changes. The world must come together to address moral concerns about the application of artificial intelligence technology. The scope of relevant international collaborations should be increased by researchers in order to uphold the noble ideal of science without borders. Although it is consistent with the current development trend of human society, the emergence of intelligent machines performing manual labor in the field of artificial intelligence technology also changes the employment structure at this time. The production and habitation needs of human society play a significant role in the development trend of artificial intelligence technology.

## 5. Conclusion

With the widespread use of artificial intelligence technology, humans' capacity to change and adapt to nature has rapidly increased, and the overall influence of nature on people has decreased. The main duties of the AI algorithm developers and controllers are condensed, and their self-regulation and self-regulation are strengthened, by strengthening the connection between the AI algorithm developers, controllers, and algorithms. In the current data recognition of machine learning, its characteristics of insensitivity to noise and good noise tolerance can be cited well, but its shortcomings are equally obvious, necessitating us to carry out technical improvement and challenging homework in constant practise. The future field of artificial intelligence will benefit from the random forest machine learning technique. Applying the art of illusion to logo design is a good way to develop a designer's ability to see the essence behind phenomena and shift perspectives. Combining optical illusion graphics with product forms creates a twofold effect by connecting one thing with another. It highlights its unique personality traits in addition to demonstrating how similar things are. In design, artificial intelligence functions more like a catalyst. On the one hand, it encourages the integration of computer science and design, and on the other, it can encourage designers' artistic inspiration. Artificial intelligence is serving as a medium for the transformation of all spheres of life. The main benefit of artificial intelligence for designers in the field of design is that it can take the place of time-consuming repetitive tasks and some traditional modes of artistic expression.

## Figures and Tables

**Figure 1:** Comparative study of human brain and machine in design work.

**Figure 2:** Model diagram of modern design products.

**Figure 3:** Design distribution data analysis diagram.

**Figure 4:** Functional data analysis diagram.

**Figure 5:** Statistical data analysis diagram.

**Figure 6:** Data map of artificial intelligence problems (1).

**Figure 7:** Data map of artificial intelligence problems (2).

**Table 1:** Design impact analysis (1).

Logo design analysis		
Type	Spoil the effect	Probability
Background	34%	36%
Modeling	57%	76%
Line	54%	56%

**Table 2:** Design impact analysis (2).

Logo design analysis		
Type	Spoil the effect	Probability
Element	32%	74%
Level	63%	25%
Degree	45%	47%

## Data Availability

The data used to support the findings of this study are available from the corresponding author upon request.
